This article has been retracted.

# Prevention of Physical Risk and Rehabilitation of Muscle Injury in Sanda Competition

**DOI:** 10.1155/2022/9486697

**Published:** 2022-07-07

**Authors:** Yong Wang

**Affiliations:** School of Physical Education and Health, Hangzhou Normal University, Hangzhou, Zhejiang, China 311121

## Abstract

*The Target*. The purpose of this study is to explore the reduction of sports injury risk and verify the effective methods and means of athlete's muscle injury rehabilitation. *Methods*. In this study, 80 sanda athletes from a university were randomly selected as subjects, and the main parts of injury of all subjects were counted. After 12 weeks of muscle injury rehabilitation intervention, the pain, acute injury, and technical and tactical evaluation levels of subjects in the intervention group and the control group were compared. *Results/Discussion*. The overall performance of the 80 subjects' basic exercise ability was at a moderate level, and there was no significant difference between male and female subjects (P >0.05). After 12 weeks of rehabilitation intervention, there was no significant difference in the scores of shoulder joint flexibility, supine straight leg raising, and trunk stable support between male and female subjects in the intervention group in more than 7 sports (P >0.05). In the control group, there were significant differences in the scores of shoulder flexibility and trunk stability of male and female subjects (*P* < 0.05). Future research should further explore the effect of muscle injury rehabilitation on effectively reducing potential sports injuries and introduce advanced and effective medical rehabilitation methods.

## 1. Introduction

It is necessary to promote health construction and improve people's health. In the development of mass sports activities, it is necessary to advocate a new trend of national fitness and promote health construction. It is necessary to improve the physical health monitoring system, develop and apply big data of national physical health monitoring, carry out exercise risk assessment, explore the relationship between exercise and health, and avoid the occurrence of exercise risks [1]. Sanda is a modern competitive sport in which two people beat each other by using offensive and defensive techniques such as kicking, hitting, and throwing in Wushu according to certain rules. It is an important part of Chinese Wushu. It not only has the characteristics of attack and defense, the practical value of fitness, and self-defense, but also has fitness and entertainment, favored by the majority of sports enthusiasts in ordinary colleges and universities. In the practice of kicking, hitting, falling, and taking and corresponding defense skills due to poor physical fitness, unscientific training and other reasons caused by sports injury risk is greater. In sanda sports, the ankle, knee, waist, hip, elbow, and wrist are prone to sports injuries. The concept of functional training was first proposed by Gray. Functional training is mainly used in the field of rehabilitation, and it is a means of functional rehabilitation, which can be understood as planned or targeted physical training to acquire certain skills [2]. Body function training is understood as a basic mode of paying attention to body posture and body movement. Training uses body integration to optimize the quality of the most basic human motor abilities. It is the strength of the movement pattern, spine, transmission chain, recovery, and regeneration, put forward a set of system optimization to improve specific movement ability training concept [3].

In the past ten years, the application of functional training in the field of sports has made a new definition of human functional training from all aspects of sports anatomy. That is, physical function training highlights the joint action of relying on nerves to control muscles, joints, and bones and mobilizing the power chain of the system, rather than only through the training of the core strength of the body can the body achieve a flexible, balanced, and efficient state. In addition, this training can strengthen the coordinated development of deep small muscles, prevent sports injuries, and improve exercise ability [4]. Existing literature [5–7] shows that most studies on sanda sports injuries remain in the following aspects, such as injury ratio, injury site, injury type, and analysis and speculation of injury causes, as well as causes and preventive measures for sports injuries. Jarl et al. studied the causes of knee joint injuries, the nature of injuries, the relationship between training years and injuries, as well as the diagnosis, treatment, and prevention, and put forward scientific and reasonable methods and suggestions for preventing knee joint injuries [8]. Rother et al. found significant differences in injury incidence among athletes of different grades [9]. Schoenfelder et al. study athlete injuries that mainly occur in competition and technical training period, and the incidence of sports injuries is relatively low during physical training period. The parts of sports injuries are mainly concentrated in head and face, wrist, ankle, and small legs. There are more than 10 kinds of sports injuries of Wushu sanda athletes. It is mainly characterized by soft tissue contusion and laceration, joint ligament injury and muscle injury [10]. Yang et al. analyzed the injury factors of Wushu sanda athletes as potential factors and direct factors and discussed the prevention measures of Wushu sanda athletes, from strengthening the physical training of Wushu athletes to improving physical reserves. Scientifically arrange the amount of exercise, strengthen the medical supervision of Wushu athletes, and improve their awareness of self-protection, so as to reduce the sports injury rate of Wushu sanda athletes [11]. At present, scholars pay attention to the sports injury probability of sanda athletes, but the related research of sanda sports injury risk prediction angle is not perfect. With the continuous development of sanda, the number of people who like sanda is expanding, so how to prevent sanda athletes and sanda enthusiasts from sports injury, reduce the risk of sports injury, prolong the life span of sports, and other related problems have posed challenges to researchers from all walks of life.

In this study, sanda enthusiasts were selected as experimental subjects, and functional motion screening tools were used to evaluate the symmetry, stability, and flexibility of the physical functional movements of sanda enthusiasts. Through the analysis of test data, it can reduce the risk value of sports injury when sanda enthusiasts complete functional movements, enhance the health awareness of sanda enthusiasts, put forward effective preventive measures and treatment means, improve the training effect, and provide reference for scientific training.

## 2. Methods

### 2.1. Design

This research takes college students' Sanda elective courses as the main research object. Through a large number of research methods such as induction, analysis, and comprehensive interpretation, the experimental data is collected for systematic analysis, and the experience of training Wushu Sanda events and injury training assistance are screened.

### 2.2. Participants

In this study, 80 people (40 males and 40 females, respectively) from Sanda Club of a certain university were randomly selected as subjects. The basic information of all subjects was age (19.13 ± 1.20 years old male and 18.50 ± 0.75 years old female), height (1.74 ± 0.04 meters male and 1.63 ± 0.04 meters female), body weight (male 66.63 ± 6.52 kg and female 58.50 ± 0.75 kg), and BMI (male 21.96 ± 1.94 and female 22.06 ± 0.99), as shown in Table 1. All the subjects are healthy and willing to participate in the study. The tester explains the detailed content of the study and matters needing attention to the subjects and signs in the informed consent form after the subjects agree.

### 2.3. Measures

There are many researches on the treatment of sports injury, such as acupuncture, massage, and cupping therapy, which are widely used in the treatment of sports injury. Traditional Chinese medicine has a good effect on sports injury. The specific method is shown in Figure 1.

Massage therapy strengthens the repair of damaged soft tissue and maintains the balance of Yin and Yang. Researchers believe that patients with medial and lateral ligament injuries of the knee joint can use acupoint massage such as Xuehai, Yanglingquan, Yinlingquan, Weizhong, Taichong, and Zusanli to effectively repair the injury 48 hours after the injury [12]. Strong stimulation press for 1 minute, lift the hamstring and gracilize tendon behind the knee, and slowly flex and extend the knee several times. Local swelling can be done by pushing, rubbing, pressing and other techniques on the periphery of swelling to reduce swelling and dredging. In the middle and late stages, you can push, rub, rub, rub and other techniques to relax the muscles around the injury and shake the knee joint.

Acupuncture has a very good effect in the treatment of muscle strain. Acupoints are usually selected by meridian acupoint selection and Asha acupoint selection. Sports teams often use acupuncture combined with electroacupuncture therapy apparatus and infrared ray, which can enhance the curative effect. The intensity of acupuncture stimulation should be limited to what the patient feels comfortable. Researchers applied the oblique needling method at Asha point to treat skeletal muscle injury. The method is to determine the insertion point, directly pierce the subcutaneous needle handle, tilt the needle body in the subcutaneous loose connective tissue layer to adjust the pointing of the tip, and then contact the surface of the muscle bundle and pierce into the muscle bundle [13]. The experimental study on the effective mechanism of oblique acupuncture at Asha acupoint has proved that it restores the muscle structure and function to normal mainly by promoting the anabolism of muscle contractile protein, so as to relieve muscle pain. Cupping therapy can improve local blood circulation and promote local metabolism and is mostly used to treat old injuries. When cupping, the size of the tank is selected according to the fat degree of the athlete's local muscles. Generally, the tank is left for ten minutes to avoid tension blisters for too long. According to the clinical practice, the internal and external use of Traditional Chinese medicine has the functions of stasis and blood circulation, meridians, and collaterals. The application of Traditional Chinese medicine must be treated according to syndrome differentiation; otherwise, the expected curative effect cannot be achieved [14]. For students with acute ankle injury, new injury medicine can be applied to the swollen area and fixed with bandage or elastic bandage on the day of injury. According to local symptoms, medication can be added or reduced dialectically. In the inflammatory swelling period, due to local bleeding stagnation, reactive inflammation and local enema occur. At this time, the treatment should be based on activating blood and removing silt, qi, and collaterals, and the new injury medicine no.2 prescription can be used. At this time, TCM should be added or reduced dialectically according to the severity of local symptoms [15]. Through the comprehensive application of a variety of physiotherapy means can effectively promote the recovery of injury. Such as fracture rehabilitation can use ultrashort wave treatment and ultraviolet treatment; soft tissue injury can be treated with ultrashort wave therapy, magnetic therapy, and infrared therapy. Extracorporeal shock wave therapy introduced recently has a good effect on bone spur and terminal disease.

### 2.4. Design and Procedures

For the purpose of the study, a randomized controlled trial was conducted on 80 subjects. The intervention lasted from April 2021 to June 2021. The score was conducted 12 weeks before intervention, and 40 people were randomly selected as the intervention group and the other group as the control group. Independent sample T test was performed on the intervention group and the control group to verify whether there was any difference in test values between the two groups. If *P* value was greater than 0.05, there was no significant difference between the two groups. After the experiment, T1 and T2 were scored by FMS test again, and test data (C1) and test data (C2) were obtained. C1 test data were compared with C2 test data to analyze whether there were significant characteristics of rehabilitation effect of muscle injury. The experimental process is shown in Figure 2.

Stage 1: During the test, the test personnel recorded the sagittal plane and frontal plane of the subjects for retrospective analysis. In the experiment, two test combinations were used for screening at the same time, and the time spent by 80 students was about 4 h. The test scores of 80 subjects and video observation during the test were analyzed to analyze the risks, and the reasons for the existence of sports injuries were summarized

Stage 2: In the formulation of corrective training plan, the functional movement training system proposed by Cook was referred to, and the key points were combined with the test results, providing an effective way for the formulation of training plan. Through repeated observation of screening videos, the causes of movement limitation, compensation, and left and right body asymmetry in the exercise of the subjects were summarized, and the muscle injury rehabilitation program was developed according to the degree of physical injury of each student

Stage 3: The rehabilitation of sports injuries of the subjects in the treatment group was statistically summarized, and regular re-examination was conducted to ensure the intervention effect

Stage 4: After the rehabilitation of the experiment, all subjects were evaluated by test score again. During the test, the tester recorded the sagittal plane and frontal plane of the subjects for retrospective analysis

### 2.5. Analysis

During training, if the subject is unable to perform normal training due to injury, he/she will consult the medical staff in the hospital to confirm whether it is an acute injury. If the injury is confirmed as acute injury, the tester will record 1 case, and finally calculate the percentage of acute injury in the total number of subjects in the rehabilitation group and the control group during the 12-week training. Before and after the 12-week intervention, 3 sanda teachers were asked to evaluate the skills and tactics of the two groups of subjects, and the testers made corresponding records according to the evaluation results.

## 3. Results and Analysis

The sanda students from several universities were selected to study their training methods, and competitions and statistics showed that sanda athletes were prone to different degrees of injury in training and competition.

### 3.1. Health Injury Risk of Sanda Athlete

Knee joint is the main joint of human body activity; its main function is flexion and extension movement and can make a little rotation movement when bending the knee. Sanda requires the use of kicking, hitting, throwing, and other actions to knock down opponents in a fast, powerful, and clever way and strive to win [16]. Therefore, the incidence of knee injuries is gradually increasing. According to the investigation of sanda students, in the total number of injuries, the average number of injuries is only one, which also shows that the injuries of sanda students are more serious. There were a lot of injuries, basically covering all parts of the body. The athletes of the sanda team are prone to different degrees of injury in training and competition, and the risk of health injury is shown in Figure 3.

As can be seen from the figure, knee joint injury caused by wrestling accounted for the largest proportion of injuries because wrestling is the most typical technical characteristics of sanda. In training and competition, players' excessive movements, fatigue, inadequate activities, incorrect technical movements, and poor psychological quality are also the causes of knee joint injury. In addition, knee joint injury caused by impact also accounts for a certain proportion. In Wushu sanda competition, the leg technique has the most points. Therefore, the use of legs is common in the competition. If both sides raise legs at the same time, both sides lack judgment, and it is easy to collide with each other. At the same time, the knee joint injury caused by fatigue and inadequate activity cannot be ignored. A good preparation is the key to a good training or competition. Athletes ignore the importance of preparatory activities at the beginning of competition or training, which will lead to weak knee muscle strength and less than optimal functional movement. Therefore, it is easy to cause various injuries of the knee joint in the process of using the action. Excessive movement, poor mental quality, poor technique, and other factors can also lead to knee injury.

### 3.2. Analysis on the Nature of Knee Joint Injury of Sanda Athletes

The experiment according to the onset of acute points, suffered a direct or indirect violence caused by injury, become acute injury, is characterized by acute onset, short course of disease, and symptoms suddenly. Chronic injury or overstrain injury caused by accumulation of micro-injury is called chronic injury or overstrain injury, which is characterized by slow onset, long course of disease and gradual onset of symptoms [17]. Acute injury is a kind of sudden injury, usually in training or competition to do a certain movement suddenly injured. There is a close relationship between chronic injury and the characteristics of sports events. One part is the inappropriate treatment of acute injury or the untimely treatment after the injury, and the early training with unhealed injuries turns into chronic after multiple injuries; the other part is the improper arrangement of training; local overtraining or overburden gradually occurs [18]. Clinical sports medicine practice shows that acute injuries are more than chronic injuries, but there is a correlation between acute and chronic injuries. Chronic injury in one site can lead to multiple acute injuries in nearby sites. Some chronic injuries result from improper treatment of acute injuries and improper transformation of post-injury training schedules. Chronic injury can become acute injury again due to sports injury. The efficacy of scientific diagnosis and treatment of acute and chronic injuries is significant [19]. Acute injury requires processing, timely, and accurate determination. Improper handling or untimely handling may lead to the development of chronic injuries in the future, affecting training and competition, and Sanda is no exception. For injuries caused at different sites, the nature of the injury is also different. The type and degree of injury of sanda athletes were statistically analyzed in the experiment, and the statistical results are shown in Figure 4.

The main types of injuries in Sanda athletes are sprains, contusions, and contusions. Through the number and proportion of injuries in different parts, it is not difficult to see that knee joint injury has become a non-negligible problem for the development of sanda. According to the degree of injury, sports injury can be divided into the following three types: “mild injury,” which can still carry out physical exercise according to the teaching and training plan after injury; those who cannot do physical exercise in accordance with the teaching and training plan within one week after the injury and need to stop or reduce local activities are classified as “moderate injury”; and completely unable to exercise for more than one week after injury is classified as “severe injury” [20]. There were 32 cases (7%) who stopped training completely, and the proportion of severe injury in different parts was 25% in waist and 25% in hand. It can be seen that the degree of sports injury of sanda athletes is mostly mild injury, accounting for 67%. The second was moderate injury, accounting for 26%. Severe injury occurred again, accounting for 7%. In the process of continuous training, the statistics of sports injury factors are shown in Figure 5.

It can be seen from the figure that the correlation coefficient between the number of injuries and the age of athletes is negative (*P* < 0.01), indicating that the number of injuries decreases with the increase of age. The correlation coefficient between the number of injuries and training years was negative (*P* < 0.01), indicating that the number of injuries decreased with the increase of training years. There was a positive correlation between the number of injuries and the level of sports (*P* < 0.01), indicating that the higher the level of sports, the fewer the number of injuries; the correlation coefficient between the number of injuries and the level of education of athletes is negative (*P* ≤ 0.01), indicating that the higher the level of education, the fewer the number of injuries; the correlation coefficient between the number of injuries and the number of games was negative (*P* < 0.01), indicating that the more games, the less the number of injuries. There was no significant correlation between the number of injury and rule change, routine competition, knowledge understanding, treatment, and height. There are many reasons for the above results, such as the continuous improvement of training level and technical level, the continuous increase of knowledge and ability, and the maturity of ideas are all related to sports injuries. The scientific arrangement of the amount of exercise is directly related to the prevention of sports injury. If the amount of exercise is too large, the body is overloaded, which is easy to cause local fatigue and damage due to the decrease of sports ability. The amount of exercise is too small, the body function cannot be excessive recovery, and cannot adapt to the large amount of exercise; the large intensity of training is also prone to injury. Accordingly, it must follow the law of motion training, be aimed at body state, undertake scientific arrangement, and raise motion achievement to reduce injury occurrence. The improvement of physical quality is closely related to the performance of special sports. The key to prevent athletes' injury is to arrange sports plan reasonably. The physical qualities required by sanda athletes are speed, strength, endurance, and the ability to hit and fight. In the process of normal training, it is necessary to strengthen the training of basic skills, pay attention to training, especially when the body and mind are tired, and pay more attention to this aspect of exercise, so as to improve the physical quality and special quality of athletes. By focusing on cultivating excellent willpower, we can lay a good foundation for systematic and high-intensity training and effectively prevent injuries.

### 3.3. Analysis of Sports Injury and Previous Injury Results

Adequate preparation before the activity can improve the excitability of the central nervous system, promote blood circulation, reduce the viscosity between muscles and ligaments, strengthen the activities of various organ systems, overcome the functional inertia of the body, and fully mobilize the energy of the athlete's body. Sanda is a direct physical combat sport. From the beginning of the competition, it requires entering the best state and giving full play to the extreme physical strength and tactics [21]. There is no short compensation period as a transition, so the preparation is more important. Preparation activity too early, too big, and too little will cause body disorders and injuries. The vulnerable parts of sanda mainly include wrist, elbow, knee, ankle, head, and waist. Special strength training should be paid attention to, and its flexibility and flexibility should be improved so that it has a certain ability to fight, so as to achieve the requirements of soft but not soft, hard but not stiff, and coordinated action. Statistics of sports injury sites are shown in Figure 6.

According to the injury status of the subjects before the 12-week exercise intervention, the injury sites were mainly concentrated in the knee joint, hip joint, ankle joint, waist, shoulder, neck, elbow joint, wrist joint, and chest, which were also the typical injury sites and types of sanda athletes. Among them, the rate of knee joint injury is the highest, accounting for 11% of the total number of injuries in both men and women. The knee joint is the main joint of the lower limbs of the human body. It consists of the patella and the fibula and can be connected to the femur and the tibia. The meniscus can be straightened and flexed, and the most fearful thing is to lean on the side when it is straightened, kicking, slapping, and hitting with both feet. This can result in a torn meniscus, damage to the lateral collateral ligament or joint dislocation, or even a fracture. Hip injuries were reported in 11% of men and 5% of women. The hip joint is an important joint that connects the body and starts the power chain. It may be due to the weak hip muscles of Sanda fans, insufficient preparation before training, technical mistakes, and large local loads. The transmission effect is poor, and the power chain eventually leads to sports damage. The ankle injury rate was 8% in men and 7% in women. The reason for the injury is that the ankle joint is connected by the tibia, fibula, calcaneus, and moment bone, which can be flexed, extended, adducted, and abducted, with a small range of motion. When twisted, pulled, or beaten by violence, dislocation, ligament tearing, and even fracture can be caused. Upper limb injuries are the waist, shoulder, elbow, and wrist joints. Due to their high flexibility, these joints are mainly the main tools for close combat of the upper limbs of the human body; from the analysis of anatomical principles, the waist includes five vertebral bodies, and different vertebral bodies are connected by intervertebral discs, ligaments, and intervertebral joints. The waist also plays a central role in the various systemic movements performed by the human body. However, due to insufficient preparation, weak local muscle strength, and other strenuous exercise, it is easy to be injured. The shoulder joint is connected by the scapula, humerus, and clavicle. It is the joint with the largest range of motion in the human body and is prone to dislocation, ligament, and muscle damage. The elbow joint is connected by the radius, ulna, and humerus and can be flexed and extended. Due to the limited range of motion, it is prone to dislocation and tearing of ligaments and muscles when high pressure is applied in the stretched state. Wrist joints, finger joints, etc. are also prone to contusion of tendons and ligaments due to incorrect force and excessively relaxed striking actions. Through the actual survey, it is found that in the subjects' daily training, 67% of people prepare for 5-10 minutes, and only 41% of people relax and arrange for 5-10 minutes. Based on the above analysis, insufficient time for preparation, relaxation, and finishing, as well as wrong movement techniques, may be the important causes of subjects' sports injuries.

## 4. Discussion

It should actively cooperate with all subjects in the experiment to complete the evaluation, arrange for specialized evaluators to carry out scientific evaluation and strictly require the objective score of each participant, and conduct evaluation of all the files of the front and the subject's archive video recording, so as to achieve the second goal. This ensures the scientific nature of the evaluation to the greatest extent. In this study, subjects were evaluated by seven motion modes: squat, hurdle, straight lunge, shoulder flexibility, active straight leg lift, trunk stability stoop, and rotation stability.

### 4.1. Analysis of Assessment Results of Different Genders before Rehabilitation Treatment

Before the 12-week intervention, 80 subjects of different genders, 40 males and 40 females, were tested. The test results of subjects of different genders are shown in Figure 7.

Before the intervention, the average score of 7 actions of 80 subjects of different genders was 15.50 for male subjects and 15.87 for female subjects, and the average score of male subjects was lower than female subjects. Independent sample *T*-test analysis was conducted on the average scores of test total scores and 7 movements of subjects of different genders, and it was found that there was no significant difference between the average scores of test total scores of subjects of different genders (*P* > 0.05), but the average scores of shoulder flexibility and straight leg lifting of females were significantly higher than those of males (*P* < 0.05). The average score of trunk stability thrust in male was significantly higher than that in female (*P* < 0.05). Both shoulder flexibility test and supine straight leg lift test can show the flexibility and flexibility of human body. Therefore, it can be inferred that the flexibility of shoulder, hip, and posterior muscle group of lower limbs of female subjects are better than that of male subjects. The body stability push-up test can show the core strength of the subject, and the strength is directly related to the power transfer efficiency of the body. High quality core capabilities can maintain stability and reflect the efficiency of energy transfer. This indicates that the core muscle strength of male subjects is superior to that of female subjects.

### 4.2. Comparative Analysis of Two Groups of Athletes with Muscle Injury Rehabilitation Intervention

After 12 weeks of muscle injury rehabilitation, 80 subjects of different genders, 40 males and 40 females, were tested. There was a significant difference between men and women in the control group before 12 weeks, but no difference after 12 weeks. The results of two gender-specific tests after 12 weeks of intervention training are shown in Figure 8.

After randomization, we count the test scores. There were no significant differences in scores for squat, hurdles, straight lunges, shoulder flexibility, supine straight leg raise, trunk stabilization support, and rotational stabilization. Independent sample *T*-test was used for statistical analysis of 7 motor test scores of male and female subjects in the intervention group and the control group, and it was concluded that after 12 weeks of intervention training, there were no significant differences in the scores of squatting, hurdle, straight lunge, shoulder flexibility, supine straight leg lift, trunk stability thrust, and rotation stability between male and female subjects in the intervention group. In the analysis of seven movements in the control group, there were still significant differences in the scores of shoulder flexibility and trunk stability of male and female subjects (*P* < 0.05). Muscle injury rehabilitation can promote the flexion and extension of hip joint in male subjects. The physical function training can improve the natural complementary ability of shoulder, thoracic vertebra and thorax, and the flexion and extension ability of hip joint in male subjects. Body function training also enhanced core muscle stability in female subjects.

### 4.3. The Number of Pains in the Two Groups before and after the 12-Week Intervention Training

In this study, sports injuries were defined as follows: After 12 weeks of rehabilitation, the subjects still needed to seek medical assistance after their training. The occurrence of acute injury in the two groups of subjects was summarized and statistically, as shown in Figure 9.

Before 12 weeks of training, 4 people in the intervention group had pain, including 2 people with knee pain, 1 person with shoulder pain, and 1 person with wrist pain. In the control group, 7 patients had pain, including knee pain in 3 patients, waist pain in 2 patients, and shoulder pain in 2 patients. After 12 weeks of rehabilitation, 2 patients in the intervention group had pain, including 2 patients with knee pain. In the control group, there were 5 people with pain, including 2 people with knee pain, 2 people with waist pain, and 1 person with shoulder pain. The reduction rate of pain in the intervention group was significantly greater than that in the control group.

## 5. Strengths and Limitations

In future physical training, Sanda athletes will transform physical training into a means of physical function training, focusing on improving the flexibility and stability of shoulder joints, hip joints, and knee joints, as well as the strength of surrounding muscles, and reducing sports injuries during physical exercise. In the future training practice, it is suggested to improve the physical performance of sanda enthusiasts by means of physical function training. The research focuses on how to increase the hip and shoulder flexibility of male sanda lovers and how to improve the stability of the core area of female sanda lovers. In the process of exercise practice, we can consider the physical function training as a supplementary exercise of physical training. The two training methods are interdependent and cannot replace either of them. In the rehabilitation measures of muscle injury, we should not only rely on a single method, means, combined with a variety of methods, in different measures to cycle treatment, so that the treatment effect is more scientific and reasonable.

## 6. Future Research

Considerations for future studies include the introduction of advanced rehabilitation treatments to reduce the risk of physical injury. The following research will establish athlete injury files, so as to share resources and conduct classified sports medicine research. For the rehabilitation of injured athletes, it is necessary to strengthen psychological adjustment, analyze the cause of injury and build self-confidence.

## 7. Implications for Practice

At present, the literature on the prevention of physical risk in sanda competition is different. This study further confirms this variable in research. The scientific arrangement of the amount of exercise is directly related to the prevention of sports injury. If the amount of exercise is too large, the body is overloaded, which is easy to cause local fatigue and damage due to the decrease of sports ability. The amount of exercise is too small; the body function cannot be excessive recovery, and cannot adapt to the large amount of exercise; large intensity of training is also prone to injury. Accordingly, it must follow the law of motion training, be aimed at body state, undertake scientific arrangement, and raise motion achievement to reduce injury occurrence. Physical fitness is not only the basis of improving the performance of special sports, but also the key to prevent athletes' injury. The physical qualities required by sanda athletes are speed, strength, endurance, and the ability to hit and fight.

## 8. Conclusion

This study analyzes the body injury sites and types of sanda athletes and puts forward the prevention measures to reduce the risk of injury. For athletes to identify the degree of muscle damage, through comparison before and after rehabilitation treatment, test the flexibility and stability of the athletes, effective understanding of basic movements, body control, sanda athletes sport ability of body flexibility and stability, etc. The results showed that the injury sites of all subjects were mainly concentrated in the knee, hip and ankle joints. The rate of knee joint injury in both male and female was 11%. Hip injury rates were 11 percent for men and 5 percent for women. The rate of ankle injuries was 8 percent for men and 7 percent for women. After 12 weeks of intervention and rehabilitation, there was no significant difference in the scores of shoulder flexibility, supine straight leg lift, and body stability stoop in the intervention group. In the control group, there were significant differences in the scores of shoulder flexibility and trunk stability.

## Figures and Tables

**Figure 1:** Rehabilitation measures for sports injury.

**Figure 2:** Flow chart of muscle injury rehabilitation test.

**Figure 3:** The cause and location of health injury.

**Figure 4:** Statistical chart of injury type and degree of sanda athletes.

**Figure 5:** Statistical chart of sports injury factors.

**Figure 6:** Statistical chart of sports injury and previous injury results.

**Figure 7:** Assessment results of different genders before rehabilitation.

**Figure 8:** 12 weeks of intervention training in two groups of different gender test results.

**Figure 9:** The occurrence of acute injury in subjects.

**Table 1:** Basic information of trainees.

	Age	Height (m)	Weight (kg)	BMI
Male	19.25 ± 0.26	1.75 ± 0.45	67.12 ± 0.56	21.34 ± 0.98
Female	18.31 ± 0.17	1.64 ± 0.36	56.53 ± 0.38	22.45 ± 0.45

## Data Availability

The data used to support the findings of this study are included within the article.
